RETRACTED

# Effect of Intelligent Medical Data Technology in Postoperative Nursing Care

**DOI:** 10.1155/2022/9681769

**Published:** 2022-08-23

**Authors:** Ninggui Duan, Guangbo Lin

**Affiliations:** ^1^School of Public Health and Management, Youjiang Medical University for Nationalities, Baise, 533000 Guangxi, China; ^2^Innovation and Entrepreneurship College, Baise University, Baise, 533000 Guangxi, China

## Abstract

Surgery is one of the larger wounds in conventional surgery, and patients often experience different pain and postural discomfort after surgery. With the ever-changing standards of medical care and patient care requirements, providing high-quality care to postoperative patients is an important measure to reduce complications and promote rapid recovery. However, in the traditional postsurgical nursing methods, there are often the phenomenon that wrong patients are connected, patient data is messy, and medicines are counted incorrectly, which directly leads to a rapid decline in nursing efficiency. In the context of the rapid development of artificial intelligence and big data, intelligent medical data analysis technology has gradually been integrated into the medical field. This paper analyzes and studies the application effect of intelligent medical data analysis technology in postoperative nursing. It is aimed at changing the traditional postoperative nursing methods and improving nursing efficiency, and it provides important suggestions for the development of postoperative nursing in the new era. Combining big data and Internet of Things technology, this paper builds a smart medical Internet of Things framework and an intelligent postoperative care system and uses machine learning algorithms to preprocess relevant medical data. The final experimental results show that the intelligent medical data analysis technology has a good effect in improving the nursing efficiency after surgery, and the nursing efficiency has increased by 6.9%.

## 1. Introduction

With the development of computer technology, nursing informatization has been put on the agenda; from the earliest manual nursing and then through the fixed nursing station, it has gradually developed to the current intelligent nursing technology. In recent years, big data and artificial intelligence have been widely used in the medical field, for example, using big data and artificial intelligence technology to diagnose and analyze patients' diseases. The application of intelligent medical data analysis technology to postoperative care is conducive to more accurate. It processes patient data more efficiently, thereby improving care efficiency and bringing quality care to patients.

With the development of modern science and technology, many research results have been achieved in the field of intelligent medical care. Guo developed a wireless smart medical tracking system. It is used to track clinical care. Test results show that the system can help medical staff to accurately identify patient information and care details [1]. Xian discussed the circuit loop technology in the intelligent medical equipment system and finally found that the technology can save a lot of power consumption in the hospital wireless power supply system and has high security [2]. Chang studied patients' willingness to receive smart medical technology at home and the specific conditions under which they could receive continuous monitoring. The results show that emphasizing trust and privacy are core patient requirements [3]. Büyükzkan developed an intelligent model for temporal classification based on horizontal visibility maps for disease diagnosis. He concluded with extensive comparative experiments on benchmark datasets, which demonstrate the superiority of the model in terms of both accuracy and efficiency [4]. Soppimath proposed a research method of telenursing assistance in emergency department based on intelligent medicine. This method provides an important reference value for the development of the hospital nursing system [5]. In the context of the development of smart medical care, the Yu and Liu teams put forward the idea of “flattening” in the integration of medical courses according to the characteristics of clinical medical information systems. It finally confirmed that the proposed educational reform program has a certain effect [6]. Elsayed applied the distributed processing technology to the intelligent medical system. The experimental evaluation results show that the technology can significantly improve the processing power and computing speed of the system [7]. The above research work on intelligent medical technology is still relatively specific, but it does not involve postoperative care.

RETRACTED

Postoperative care is an indispensable part of patients after surgery, and many scholars have also conducted research on postoperative care. Ahmad discussed the use of Arden grammars to test the feasibility of coding large postoperative care plans. It turns out that the Arden grammar is able to encode all necessary functions of a care plan [8]. Jones proposed a list-based tool to avoid bias during patient examination. The tool was found to significantly reduce serious errors in the patient checklist [9]. Roeleveld analyzed the effect of tumescent liposuction in methods to optimize postoperative care of patients. Results showed that the swelling technique significantly improved postoperative comfort and accelerated recovery time [10]. Chan proposed a multimodal postoperative nursing monitoring method and finally proved the important value of multimodal monitoring in neurocritical care patients. It helped to provide optimal treatment for patients based on individual pathophysiological changes [11]. Tzer discussed the importance of diet in postoperative care of patients after pancreatic surgery. Finally, he found that giving patients a diet high in fat and enzymes could prevent a series of complications after pancreatic surgery in patients [12]. Nguyen analyzed the importance of postoperative care of patients after cataract surgery and finally found that the use of protective eyewear after simple cataract surgery can avoid ocular complications [13]. Nelson explored the interrelationship between intensive care postoperative systems and perioperative care activities. His final finding was that the use of nonclinical methods could provide insight into the operation of the perioperative care system, enabling the identification and elimination of bottlenecks in patient flow [14]. These studies on postoperative care are relatively detailed, but they have not been applied to intelligent medical data analysis technology.

In order to change the traditional postoperative care model and improve the quality and efficiency of care, this paper applies the intelligent medical data technology to postsurgical care. An intelligent nursing system is constructed by combining technologies such as the Internet of Things and artificial intelligence [15]. In this paper, relevant algorithms are used to process and analyze the medical data in the system. Finally, the experimental test verified that the intelligent medical data technology can achieve good results in the nursing quality and nursing efficiency of postoperative nursing. It provides an important reference value for the improvement and upgrading of postoperative care.

## 2. Intelligent Medical Data Framework

In the context of the rapid development of the Internet of Things, medical big data has been widely used in different medical environments [16]. The Internet of Things is an extension and expansion network based on the Internet. It is a huge network formed by combining various information sensing devices with the Internet to realize the interconnection of people, machines, and things at any time and any place. At present, many scholars have realized the continuous monitoring of patients' heartbeat, blood pressure, blood sugar level, and body temperature through IoT technology. It uses this data for disease diagnosis and clinical care. Typically, these medical big data come from sensors worn by patients who support IoT technology.

RETRACTED

IoT devices continue to generate massive amounts of structured and unstructured data often referred to as big data [17]. In the medical field, data security and data analysis are key to the medical system. In order to better process and analyze the data, this paper applies the Internet of Things to the medical big data system.  Figure 1 is an intelligent medical data analysis framework based on the Internet of Things. The framework mainly includes five parts: wearable devices, sensors, controllers, actuators, and various smart terminals. The implementation process: it first provides patients with smart wearable devices and then collects data from the wearable devices (the acquisition process includes data transmission and signal reception of sensors, controllers, and actuators). Then, these data will be sent to various smart terminals in time. In the end, the doctor or nursing staff will arrange the follow-up nursing work according to the patient data on the terminal [18, 19].

## 3. Application of Intelligent Medical Data Technology in Postoperative Nursing

Intelligent medical data analysis technology can use mobile devices to collect and analyze data. It can also use widescreen projection equipment to display and promote the data. It helps nurses to fully understand the patient's postoperative diagnosis and treatment information and then formulate a scientific nursing plan for the patient.

### 3.1. Postsurgery Intelligent Nursing System

Usually, postsurgery nursing work includes fluid infusion, postoperative sign collection, admission and discharge, treatment implementation, and daily care [20]. This paper uses intelligent medical data analysis technology to rationally optimize traditional nursing work, thereby improving the quality and efficiency of postoperative nursing work, meeting the nursing needs of patients, and dealing with postoperative emergencies (such as postoperative complications).  Figure 2 is a schematic diagram of an intelligent postsurgery nursing system based on medical data analysis. Overall, the system is divided into display part, application part, and data part from top to bottom. The display part mainly uses the logic functions provided by the application part to export relevant data to different display platforms and then interact with nursing staff. The application part, also called the business logic part, is the core of data processing, and most business logic is represented in this part. The various interactive information in the display part is accessed to the database through the analysis and processing of the application part. The data part accesses the underlying database through the data access tool provided by the system, thereby providing data support for the application part.

RETRACTED

The application part and the presentation part are interconnected. The application part mainly includes four modules: nursing knowledge base, nursing plan, nursing information reminder, and ward system. The display part is various intelligent terminals. The nursing knowledge base is the core of the application part, and the knowledge files are stored in the form of archives. It is also displayed using terminal equipment such as electronic whiteboards, tablet computers, mobile terminals, and LCD TVs. For example, the information displayed by the nursing staff on the electronic whiteboard: brief introduction of the ward (including the display of the number of admissions and discharges and the distribution of beds for critical care, primary care, secondary care, and tertiary care and display them in images), workload statistics (including body temperature, intramuscular injection, skin test, static push, and other workload statistics), nursing plan (including all-day plan, executed plan, and unexecuted plan), reminder information (including crisis value reminder), basic patient information (including bed number, name, gender, age, cost details, and nursing level), patient characteristics (surgery patient, level of care), etc.

### 3.2. Segmentation of Intelligent Nursing System

As shown in Figure 3, the intelligent nursing system includes six components: postoperative patient management, doctor's order management, nursing document management, ward management, configuration management, and nursing management. Postoperative patient management is divided into basic patient information management, status management, sign management, hospital admission management, doctor order management, and reminder management related to patients. Medical order management is divided into medical order query statistics, medical order classification management, execution management, medical order data update management, etc. Nursing document management is divided into document creation, filling, updating, changing, printing, etc. Ward management is divided into ward operation management, nurse management, and drug management. Configuration management mainly includes server configuration, computer configuration, and configuration of portable terminal equipment. It is a series of measures to control and standardize software products and their development process and life cycle through technical or administrative means. The goal of configuration management is to record the evolution of software products and ensure that software developers can obtain accurate product configurations at all stages of the software life cycle [21, 22].

RETRACTED

The specific processing process of postoperative nursing work is shown in Figure 4, which is divided into postoperative patient dynamics, department workload, nursing notification, and shift scheduling. The dynamic part of postoperative patients is to calculate the number of admissions and discharges of patients, which is reflected in the admissions and discharges of patients in each department every day. On the other hand, according to the patient's nursing level and statistical quantity, the patient's condition in each department can be fully grasped. The workload of the department is a statistical analysis of the workload of the department according to the condition of the postoperative patients, medical resources, and the workload of the nurse's doctor's order, and the results of the statistical analysis are checked. Nursing notice is that the nursing department publishes the content of notices and announcements to various departments and subordinate medical and nursing units and distributes them to relevant personnel in the form of messages. The scheduling statistics are divided into the statistics of historical shifts and the statistics of this week's shifts.

The execution of doctor's orders is the core part of postoperative nursing work, and most of the work of nursing staff is carried out in accordance with the execution of doctor's orders [23]. As the most important step in nursing work, the execution of doctor's orders is more complicated. Taking the infusion doctor's order as an example, it requires four steps: checking the medicine placement, checking the dispensing, executing the doctor's order, and performing the check. The specific process is shown in Figure 5. Among them, the drug check should analyze the total number of valid prescriptions for each patient in the hospital and the number of prescription bottles executed by each patient at the same time. In the dispensing check, it is necessary to check whether the number of prescriptions of the patient corresponds to the infusion bottle and remind the nursing staff to check the validity period and dosage of each bottle of infusion medicine.

## 4. Postoperative Nursing Data Processing Algorithm

In order to further improve the role of intelligent medical data analysis technology in postsurgical care, this paper uses classification technology in machine learning to process relevant nursing data. Generally speaking, text classification systems can be divided into two categories according to the different methods of obtaining classification information: classification systems based on machine learning and classification systems based on knowledge engineering [24]. Text classification is a method of using a computer to automatically classify and mark a text set (or other entities or objects) according to a certain classification system or standard. Due to the complexity of medical data and the large amount of information, this paper adopts a text classification method based on statistical machine learning when classifying texts.

RETRACTED

### 4.1. Principal Component Analysis

Principal component analysis, also known as principal component analysis, is a statistical technique based on dimensionality reduction methods [25]. The use of principal component analysis can play a role in reducing the dimension and synthesize multiple indicators into a few independent comprehensive indicators (i.e., principal components), each of which can reflect most of the information of the original variables, which contains nonrepetitive information.

#### 4.1.1. Data Standardization

(1) $$\begin{array}{c} Z_{ij}=\frac{x_{ij}-{\bar{x}}_{j}}{S_{j}},i=1,2,\cdots ,n,j=1,2,\cdots ,p. \end{array}$$

Among them, ${\bar{x}}_{j}=\sum_{i=1}^{n}x_{ij}/n$, $S_{j}^{2}=\sum_{i=1}^{n}{\left(x_{ij}-{\bar{x}}_{j}\right)}^{2}/\left(n-1\right)$.

#### 4.1.2. Calculate the Correlation Coefficient Matrix

(2) $$\begin{array}{c} R={\left[r_{ij}\right]}_{p}xp=\frac{Z^{T}Z}{n-1}. \end{array}$$

Among them, *r*_*ij*_ = ∑*Z*_*kj*_*Z*_*kj*_/(*n* − 1), *i*, *j* = 1, 2 ⋯ , *p*.

#### 4.1.3. Solve the Matrix to Determine the Number of Principal Components

(3) $$\begin{array}{c} \left|R-\lambda I_{p}\right|=0, \end{array}$$

(4) $$\begin{array}{c} \frac{\sum_{j=1}^{m}\lambda_{j}}{\sum_{j=1}^{p}\lambda_{j}}\geq 0.85. \end{array}$$

Solve formula (3) to obtain the characteristic root of the formula, determine the value of *m* in formula (4), find the formula *Rb* = *λ*_*j*_*b* of each *λ*_*j*_, *j* = 1, 2, ⋯, *m*, and obtain the characteristic vector *b*_*j*_^*o*^.

#### 4.1.4. Principal Component Generation

(5) $$\begin{array}{c} U_{ij}=Z_{i}^{T}b_{j}^{o},j=1,2,\cdots ,m. \end{array}$$

In the formula, *U*_1_, *U*_2_, and *U*_3_ are the first, second, and third principal components, and so on, *U*_*m*_ is the *m*-th principal component, *U*_*ij*_ represents the principal component, and *Z*_*i*_^*T*^ represents the covariance variable.

#### 4.1.5. Principal Component Evaluation

The *m*-th *U*_1_, *U*_2_,…, *U*_*m*_ principal components are first weighted and then aggregated to obtain the score, in which the contribution rate of variation is the weighted value.

### 4.2. Support Vector Machine

Support Vector Machine (SVM) is a data mining technique that uses a simplified approach to solving problems related to machine learning.

RETRACTED

According to the given training set, *O* = {(*a*_1_, *b*_1_), (*a*_2_, *b*_2_), ⋯, (*a*_*l*_, *b*_*l*_)} ∈ (*A* × *B*)^*l*^.

*a*_*i*_ ∈ *A* = *R*^*n*^, *A* are the input space, the input space *a*_*i*_ is composed of *n* attribute features, and *b*_*i*_ ∈ *B* = {−1, 1}, *i* = 1,…, *l*; the classification function is used by finding a real-valued function *R*^*n*^ on *g*(*a*), that is,

(6) $$\begin{array}{c} f\left(a\right)=\mathrm{sgn}\left(g\left(a\right)\right). \end{array}$$

Consider the training set *O*, if *ω* ∈ *R*^*n*^, *k* ∈ *R*, and *ε* > 0, make the subscript *i* of all *b*_*i*_ = 1 have (*ω* · *b*_*i*_) + *k* ≥ *ε*, and make the subscript *i* of *b*_*i*_ = −1 have (*ω* · *b*_*i*_) + *k* ≤ −*ε*, and then, *O* is linearly separable, that is, the corresponding classification problem is linearly separable.

Denote the two types of sample sets as {*M*^+^ = {*a*_*i*_|*b*_*i*_ = 1, *a*_*i*_ ∈ *T*}} and {*M*^−^ = {*a*_*i*_|*b*_*i*_ = −1, *a*_*i*_ ∈ *O*}}. Define the convex hull conv(*M*^+^) of *M*^+^ as

(7) $$\begin{array}{c} \text{conv}\left(M^{+}\right)=\left\{a=\overset{N_{+}}{\underset{j=1}{\sum }}\lambda_{j}a_{j}\left|\overset{N_{+}}{\underset{j=1}{\sum }}\lambda_{j}=1,\lambda_{j}\geq 0,j=1,\cdots ,N^{+},a_{j}\in M^{+}\right.\right\}. \end{array}$$

*M* ^−^ has convex hull conv(*M*^−^) as

(8) $$\begin{array}{c} \text{conv}\left(M^{-}\right)=\left\{a=\overset{N_{-}}{\underset{j=1}{\sum }}\lambda_{j}a_{j}\left|\overset{N_{-}}{\underset{j=1}{\sum }}\lambda_{j}=1,\lambda_{j}\geq 0,j=1,\cdots ,N^{-},a_{j}\in M^{-}\right.\right\}. \end{array}$$

First, demonstrate its necessity.

If *O* is linearly separable and *M*^+^ = {*a*_*i*_|*b*_*i*_ = 1, *a*_*i*_ ∈ *O*}, *M*^−^ = {*a*_*i*_|*b*_*i*_ = −1, *a*_*i*_ ∈ *O*} is linearly separable, it can be known that there are hyperplanes *H* = {*a* ∈ *R*^*n*^ : (*ω* · *a*) + *k* = 0} and *ε* > 0 such that

(9) $$\begin{array}{c} \text{conv}\left(M^{-}\right)=\left\{a=\overset{N_{-}}{\underset{j=1}{\sum }}\lambda_{j}a_{j}\left|\overset{N_{-}}{\underset{j=1}{\sum }}\lambda_{j}=1,\lambda_{j}\geq 0,j=1,\cdots ,N^{-},a_{j}\in M^{-}\right.\right\}. \end{array}$$

And each point on the convex hull of the positive class point set and each point in the convex hull of the negative class point set can be expressed as

(10) $$\begin{array}{c} a=\overset{N_{+}}{\underset{i=1}{\sum }}\alpha_{i}a_{i},\\ \hat{a}=\overset{N_{-}}{\underset{j=1}{\sum }}\beta_{i}{\hat{a}}_{j}. \end{array}$$

Among them, *α*_*i*_ ≥ 0, *β* ≥ 0, ∑_*N*_+__^*N*_+_^*α*_*i*_ = 1, and ∑_*j*=1_^*N*_−_^*β*_*i*_ = 1.

Therefore, it can be obtained

(11) $$\begin{array}{c} \left(\omega \cdot a\right)+k=\left(\omega \cdot \overset{N_{+}}{\underset{i=1}{\sum }}\alpha_{i}a_{i}\right)+k=\overset{N_{+}}{\underset{i=1}{\sum }}\alpha_{i}\left(\left(\omega \cdot a_{i}\right)+k\right)\geq \varepsilon \overset{N_{+}}{\underset{i=1}{\sum }}\alpha_{i}=\varepsilon >0,\\ \left(\omega \cdot \hat{a}\right)+k=\left(\omega \cdot \overset{N_{-}}{\underset{j=1}{\sum }}\beta_{j}{\hat{a}}_{j}\right)+k=\overset{N_{-}}{\underset{j=1}{\sum }}\beta_{i}\left(\left(\omega \cdot {\hat{a}}_{j}\right)+k\right)\geq -\varepsilon \overset{N_{+}}{\underset{i=1}{\sum }}\alpha_{i}=-\varepsilon <0. \end{array}$$

It can be seen that the convex hulls of the positive and negative point sets lie on both sides of (*ω* · *a*) + *k* = 0, so the two convex hulls are separated.

RETRACTED

Then, prove its sufficiency.

Assume that the convex hulls of the two point sets *M*^+^ and *M*^−^ are separated. Since both convex hulls are closed convex sets and bounded, we can know that there is a hyperplane *H* = {*a* ∈ *R*^*n*^; (*ω* · *a*) + *k* = 0} that strongly separates the two convex hulls through the strong separation theorem of convex sets. That is, there is a positive number *ε* > 0 so that any points *a* and $\hat{a}$ of the *M*^+^, *M*^−^ convex hull have

(12) $$\begin{array}{c} \left(\omega \cdot a\right)+k\geq \varepsilon ,\\ \left(\omega \cdot \hat{a}\right)+k\leq -\varepsilon . \end{array}$$

Obviously, for any *a*_*i*_ ∈ *M*^+^, there is (*ω* · *a*_*i*_) + *k* ≥ *ε*, and for any *a*_*i*_ ∈ *M*^−^, (*ω* · *a*_*i*_) + *k* ≤ −*ε*, there is *O*. Through the definition of linearly separable training set, we can know that EE is linearly separable.

Since the hyperplane can be written in the form of (*ω* · *a*) + *k* = 0 in space *R*^*n*^, the same hyperplane is obtained by multiplying the parameter (*ω*, *k*) by any nonzero constant, and then, the condition is satisfied

(13) $$\begin{array}{c} b_{i}\left(\left(\omega \cdot a_{i}\right)+k\right)\geq 0,\;i=1,\cdots ,l,\\ \underset{i=1,\cdots ,l}{\min}\left|\left(\omega \cdot a_{i}\right)+k\right|=1. \end{array}$$

If the samples of the training set are linearly separated, there exists a canonical hyperplane (*ω* · *a*) + *k* = 0; it lets

(14) $$\begin{array}{c} \left(\omega \cdot a_{i}\right)+k\geq 1,b_{i}=1,\\ \left(\omega \cdot a_{i}\right)+k\leq -1,b_{i}=-1. \end{array}$$

### 4.3. Multilayer Perceptron

Multilayer perceptron is a multilayer neural network model, which is a network formed by adding hidden layers to a neural network composed of single-layer neurons.  Figure 6 is the layout diagram of the multilayer perceptron structure; a fully connected network consists of input layer, hidden layer, and output layer.

Input layer: it has the function of transferring information, and its activation function is similar to the identity function.

RETRACTED

Hidden layer: the first hidden layer is fully connected to the input layer, and the second hidden layer is fully connected to the first hidden layer. The third hidden layer is fully connected to the second hidden layer, and the output function is *f*(*W*^(1)^*a* + *k*^(1)^). *W*^(1)^ represents the weight, *k*^(1)^ represents the bias value, and the function *f* usually uses the sigmoid function:

(15) $$\begin{array}{c} \text{sigmoid}\left(a\right)=\frac{1}{1+e^{-a}}. \end{array}$$

Output layer: the output layer is fully connected to the third layer, the number of output lines is softmax(*W*_2_*a*_1_ + *B*_1_), and *a*_1_ represents the output *f*(*W*_1_*a* + *k*_1_) of the hidden layer.

Combining the above three-layer functions, the MLP function softmax can be obtained:

(16) $$\begin{array}{c} f\left(a\right)=G\left(k^{\left(2\right)}+W^{\left(2\right)}\left(s\left(k^{\left(1\right)}+W^{\left(1\right)}a\right)\right)\right). \end{array}$$

In the formula, *W*^(1)^, *k*^(1)^, *W*^(2)^, and *k*^(2)^ are the parameters, and these parameters are finally determined by the gradient descent algorithm.

## 5. Application Result of Intelligent Medical Data Technology in Postoperative Nursing

It first tested the results of machine learning methods on postoperative care data, a text classification problem. Set the number of learning samples to 1000. For the postoperative care data of three surgical procedures: ophthalmology, orthopedics, and thoracic surgery, the selected test set contains 300, 400, and 300 items. In order to avoid the imbalance of the dataset, the test set is randomly divided. Similarly, the softmax function is used as the text classification function, and the training method adopts stochastic gradient descent (SGD), and the obtained test results are shown in Table 1.

From the data in Table 1, it can be seen that the highest accuracy rate is 0.93, and the highest recall rate is 0.95, which is close to 0.96. The highest *F*1 value reached 0.96, and the recall rate and the lowest *F*1 value also reached 90%. Overall, the classification effect of machine learning methods in postoperative care data is still good, and the best classification effect is the postoperative care of orthopedic surgery.

In order to verify the application results of intelligent medical data analysis technology in postoperative nursing, the wound healing degree of 1000 surgical patients in a hospital within 10 days was selected as the experimental object under the postoperative nursing method proposed in this paper. The degree of healing is divided into three categories: relatively good, general, and poor. The experimental results are shown in Figure 7.

RETRACTED

It can be seen from the bar graph in Figure 7 that in the first five days, the number of people with normal wound healing and poor wound healing has always been relatively large. The number of people with better wound healing is lower. This is because the patient's wound healing requires a process just after surgery. However, with the blessing of postoperative care, the number of people with better wound healing in the first five days has been on the rise. After five days, the number of people with better wound healing began to increase dramatically. The number of wound healing average and poor wound healing also slowly decreased. This also suggests that postoperative care plays an important role in the healing of a patient's wound.

Figure 8 shows the comparison of the processing volume and error rate of nursing staff in processing postoperative patient data under the postoperative care system combined with intelligent medical data analysis technology (hereinafter referred to as the intelligent postoperative care system) and the traditional postoperative care mode picture. As can be seen from Figure 8, with the support of the intelligent postoperative care system, the amount of data processed by the nursing staff has always been higher than that of the traditional nursing model. On the sixth day, the processing capacity was as high as 628, while the traditional mode was only more than 300. In terms of error rate, although both modes have fluctuation trends, the intelligent postoperative care system is generally higher than the traditional postoperative care mode.

Postsurgery care includes not only disease care but also normal physiological needs and physiological performance as part of postoperative care. In order to better understand the postoperative recovery status of postoperative patients under the intelligent nursing system, this paper compared the sleep quality and dietary status of postoperative patients in two modes within eight weeks. The specific scoring standard is 0-10 points, and the test results are shown in Figure 9.

Overall, the sleep quality and dietary status of patients after surgery fluctuated greatly within eight weeks. But with the help of postoperative care, sleep quality and diet improved. In particular, the score of the intelligent nursing system is still very high, and the score reflects the effect of the two nursing modes in postoperative care. Obviously, the smart nursing system works better.

In order to further verify whether the intelligent medical data analysis technology can achieve good results in postoperative nursing, the patient's praise and nursing efficiency of the two postoperative nursing modes in 12 months were compared. Among them, the favorable rating of traditional nursing mode is marked as favorable rating A, and the favorable rating of intelligent nursing mode is marked as favorable rating B. Similarly, the nursing efficiency is marked as nursing efficiency A and nursing efficiency B, respectively, and 1 is the best value for the favorable rating and the efficiency value. The specific test results are shown in Figure 10, in which the bar graph represents the favorable rating and the line graph represents the nursing efficiency. As can be seen from Figure 10, the intelligent postoperative care system has always been in a leading position in terms of praise, and the praise is high, always between 0.85 and 0.95. In terms of nursing efficiency, although both modes fluctuate, in general, the postoperative nursing efficiency of the intelligent postoperative nursing system has been higher than that of the traditional model, and the nursing efficiency is 6.9% higher. This also confirms that intelligent medical data analysis technology can achieve good results in postoperative care.

RETRACTED

## 6. Conclusion

To sum up, differences in postoperative care systems will affect the recovery process of patients, as well as the data results of intelligent medical care. In the process of surgical treatment, superb technical operation and correct surgical plan are the keys to whether patients can regain their health. After the operation is completed, it is essential to provide high-quality and efficient postoperative care for the patient. With the acceleration of social progress, the traditional postoperative care model has been unable to meet the postoperative needs of patients. In the context of the rapid development of big data and artificial intelligence, intelligent medical data analysis technology provides technical support for the change and upgrade of postoperative care models. It also plays an important role in improving the efficiency of postoperative care and promoting the development of nursing work.

## Figures and Tables

**Figure 1:** IoT-based intelligent medical data analysis framework.

**Figure 2:** Intelligent nursing system after surgery.

**Figure 3:** Main functions of the intelligent nursing system.

**Figure 4:** Postoperative care work.

**Figure 5:** Execution process of a doctor's order.

**Figure 6:** Multilayer perceptron structure.

**Figure 7:** Degree of wound healing in surgical patients within 10 days.

**Figure 8:** Postoperative patient data processing volume and error rate.

**Figure 9:** Sleep quality and dietary status of postoperative patients in two modes.

**Figure 10:** Patient praise and nursing efficiency of the two postoperative care modes.

RETRACTED

**Table 1:** Nursing data after three surgical procedures.

Surgery category	Accuracy	Recall	*F*1
Ophthalmology	0.9235	0.9133	0.9052
Orthopedics	0.9287	0.9579	0.9500
Thoracic surgery	0.9324	0.9086	0.9617

## Data Availability

This article does not cover data research. No data were used to support this study.
